# A Crop Growth Prediction Model Using Energy Data Based on Machine Learning in Smart Farms

**DOI:** 10.1155/2022/2648695

**Published:** 2022-10-12

**Authors:** Saravanakumar Venkatesan, Jonghyun Lim, Yongyun Cho

**Affiliations:** Department of Artificial Intelligence Engineering, Sunchon National University, Suncheon-si, Jeollanam-do, Republic of Korea

## Abstract

In the recent past, the agricultural industry has rapidly digitalized in the form of smart farms through the broad usage of data analysis and artificial intelligence. Commonly, high operating costs in a smart farm are primarily due to inefficient energy usage. Therefore, accurate estimation of agricultural energy usage and environmental factors is considered as one of the significant tasks for crop growth control. The growth sequences of crops in agricultural environments like smart farms are related to agricultural energy usage and consumption. This study aims to develop and validate an algorithm that can interpret the crop growth rate response to environmental and solar energy factors based on machine learning, and to evaluate the algorithm's accuracy compared to the base model. The proposed model was determined through a comparative experiment of three representative machine learning techniques, which are random forest (RF), support vector machine (SVM), and gradient boosting machine (GBM), considering the energy usage for environmental control is highly associated with the paprika crop growth. Through the experiment performance with real data gathered from a paprika smart farm in South Korea, the multi-level RF can effectively predict paprika growth with an accuracy of 0.88, considering data analysis of factors that use solar energy. As a result of the experiment with the suggested model, the growth factors such as leaf length, leaf width, and environmental factors were found. Furthermore, the proposed algorithm can contribute to the development of applications through analysis of the crop growth big data for various plants in agricultural environments such as a smart farm.

## 1. Introduction

Sustainable agriculture is extremely important and closely related to smart farming because it improves the environmental sustainability and resource based on which agriculture relies while still meeting simple human food requirements [1].  Figure 1 shows an architecture of a smart farm to challenge the sustainability of future agriculture [2]. As shown in Figure 1, all the parts in a smart farm are intricately connected with energy. So, all processes for crop growth use energy and need observation for efficient energy usage.

Paprika (Capsicum annuum L) production observation is necessary for increasing the growth of greenhouse paprika. It is one of the most widely grown vegetables in the world and one of the most important vegetable crops for vitamins and human nutrition [1].

Paprika growth observation is essential for optimizing administration and maximizing the production of paprika in a greenhouse. Leaf growth and leaf width are critical factors for crop growth. The linear classification methods for finding attributes related to crop production may be relatively accurate [3]. The paprika growth data gained from sensors and devices can quantify production-related attributes. The variable-enhanced binary models such as SVM, RF, and GBM vector analysis classification methods may be good solutions for crop growth forecasts. The RF model could well estimate the paprika leaf growth and solar energy value that may relate to the relationship between sensors. Computer-sensor-based rules have aided the growth of paprika over other processes for estimating development-related attributes, which have yielded promising results [4]. This research area has two types: first, the models use crop training data; second, the models get energy sensor data in the field, where randomness because of non-linear data and cluttered environments was unavoidable, and the aim is to sectionalize sensor data to retrieve attributes, theoretically lowering the output [5]. The models depend on training and testing of data-driven characteristics, which solve the procedure's complexity. The solution's generality of non-linear dataset efficiency is weak. Researchers should create more linear powerful data. Machine learning attitude will directly take an environmental dataset as input and learn to construct feature representations for futuristic techniques. Machine learning can achieve higher accuracy than traditional approaches with enough datasets [6]. This research has also been used to determine which environmental factors are the most important in the growth of crops. The study's major focus is to assess and compare the performance of the two beds using the linear classification method and machine learning, in which the correlation of paprika growth was identified by leaf width, environmental factors, and solar energy [7]. The traits of SVM, RF, and GBM models were used to determine the relationship between the growth and environmental characteristics of greenhouse paprika. This paper analyzed the expected data using machine learning with sensors to monitor the growth of similar attributes of paprika.

The greenhouse observation system is intended to meet the need for remote greenhouse monitoring and control [8]. In this article, gateway architecture was implemented which denotes the system's core. In the greenhouse monitoring and control system, the IoT gateway is a joint point of the public network and wireless sensor network [9]. Its role is to realize big data collection, uploading, and processing of remote user control information [10, 11]. The gateway was built using the modularization process, which increased compatibility and allowed it to meet the better demands of a complex smart farm climate.

The greenhouse readings are wirelessly distributed from routing nodes to a central monitoring facility in the base station [12]. Messages can travel across several nodes to reach the base station, depending on the distance between the node and the base station. To read, archive, and monitor the collected data, the base station is linked to the host device running in mote view. In wireless network arrangement, the data measurement subsystem, and the base station with its graphical interface are involved with three major subsystems. MICAz wireless motes programmed in nesC are used in this wireless networking platform, and data is transmitted to a central database using an 802.15.4 wireless network [13]. Different network topologies were used to measure the stability of the deployed network. The main interface for wireless networks and other applications is Xserve. Xserve's key capabilities provide data routing to and from the mesh network, as well as higher-level services to parse, transform and process data as it travels through the mesh and external applications.

TinyOS is a free and open-source operating system for wireless sensor networks. It has a component-based architecture, which allows fast creativity and execution while reducing code size, which is essential due to the extreme memory restrictions that sensor networks impose. TinyOS comes with a component library that specifically includes network protocols, distributed services, sensor driver, and data acquisition software which are used [13]. TinyOSs' event-driven execution paradigm allows for fine-grained power control and the scheduling versatility required by the unpredictability of wireless networking and physical environment interfaces. There are three computational principles of components: instructions, events, and functions. Inter-part coordination is handled by commands and events, while intra-part concurrency is expressed by assignments. Using the nesC programming language, the wireless modules are coded with application specific TinyOS code.

Figure 2 shows the components that make up the IoT software subsystem [12]. On the MICAz modes, data is collected through sensors. The data was collected and analyzed before being sent to the MIB 250 service support platform, which was used for research and operations management. The operation is then passed to the greenhouse monitoring system module in charge of establishing relations with customers through the mote view interface or another IoT-based web/mobile customer interface [14]. User verification, server entry, data query, and update are the three aspects of the web application program that use ADO.NET to access the database.

### 1.1. Review

Recently, using big data-analysis skills, many scientists have examined the agriculture environmental and IoT-based sensor prediction problems. Through these research tries on the paprika growth patterns, several statistical and machine learning methods were developed. Because the data mining process can be hampered due to the high dimensionality and size of large datasets, the studies for an efficient feature selection have been researched as an important pre-processing step to minimize dataset dimensionality for the most informative features and classification accuracy optimization [15]. The industrial Internet of Things, sensor networks, cloud computing, and big data integration have recently been established as critical aspects in ICT-based agriculture and cloud computing systems are being built to store and process data efficiently in the industrial Internet of Things, and data analytics techniques are used to extract useful information from the vast data in the industrial Internet of Things [16]. The study using methods to address concerns on performance, multilayer perception, support vector machine, and other techniques has been used in recent work [17]. The analysis study using the models reveals total water use, plant growth rates, and the timeframe for harvesting produced by monitoring variables such as luminosity, humidity, temperature, and water use. The device allows for automatic monitoring of the greenhouse's indoor atmosphere through an irrigation system or temperature control, as well as the presentation of the main outline of agricultural product internal traceability from seed to the final product. While information and communication systems are commonly used incorporating common sense or experience into decision-making remains difficult. One research for semi-autonomous greenhouse control aims to create rules that combine the advantages of an accomplished grower and powerful machinery using information graphs and semantic analysis as a foundation [18]. Because capsicum annuum L. is so vulnerable to water shortages and is usually grown under irrigation, deficit irrigation strategies for paprika could boost efficiency, make mechanical harvesting easier, and save water at the same time. Five varied sizes of TS a were used in this analysis for improved and more reliable model evolutions of solar energy forecasting: 50%, 60%, 70%, 80%, and 90%. Such statistical indexes of the various data selections are calculated from k-fold in two training sets accuracy, precision, and kappa [19]. The research presenting the findings revealed that the RF model has excellent prediction accuracy for all training data collection values. R2 was observed to have an average value of more than 0.88. The evaluation efficiency of both SVM and GBM models would be increased by reducing the size of the training selection [20]. Literature talks about the leaf length, distance, area, and shape ratio leaf length/width, as well as a node number, were measured ten months after transplanting paprika leaves. The construction of regression equations was aided by leaf length and width measurement among them and the equations with high correlations were selected and used in validation [21]. Literature using the leaf length and width measurements, as well as the node number, was used to train an AI system GBM, SVM, and RF. When a regression equation based solely on leaf area and distance was used to measure leaf areas, the precision declined when the equation was applied separately to the upper and lower leaves. LeNet is based on neural network architecture for leaf area index in root-based paprika growth. The authors used data from an open-source local greenhouse, in which the growth factor was measured every 2 weeks and the model was implemented with a neural network and leaf area [22]. This study is to evaluate and compare the linear classification approaches and machine learning models with each other for the prediction performance of paprika growth considering environmental factors and solar energy data in the two beds [23]. Literature using [24] eight environmental factors from the days following transplanting and two crop development traits made up the algorithm, which produced weekly crop growth rates as an output. The data gathered from a commercial greenhouse were used to validate the RNN-based crop growth rate estimate method. Literature presents [25] that the success of agriculture and related businesses in the US is essential for long-term economic growth and prosperity. By carefully deciding on the ideal crops and putting in place supportive infrastructure, agribusiness crop yields may be boosted. When creating agricultural projections, various elements such as the weather, soil fertility, water availability, water quality, crop pricing, and others are taken into account. Machine learning is essential for predicting agricultural production since it can forecast crop yield based on variables like location, weather, and season. This study is to better understand the relationship between greenhouse agriculture output and various predictors. We also investigate the efficacy of various machine learning models SVM, GBM, and RF in predicting paprika growth, environment, and energy. The studies mentioned above provide information on previous research on paprika leaf growth, width, and energy prediction in various smart farm modes. Such research reflects the need to predict paprika growth to improve different applications. Many techniques are used to forecast the length of an environmental factor, but data mining techniques can be an effective method for providing adequate performance prediction.

## 2. Materials and Method

In this research, we have used the greenhouse paprika data in the year October to December 2019 and January to July 2020 total of 9 months. The paprika data is based on leaves number, leaves width, environmental factors, solar energy data, etc., We collected data from a local paprika greenhouse production in Korea. We have given a full expansion of the site and greenhouse agriculture in this study. It provides growth and energy properties in the additional material and variable in Table 1.

The data was gathered from the two independent rows, R1 and R2, on a paprika farm. All the samples of plant growth-related 3884 and environment-related 48230 were collected.  Figure 3 shows solar energy entirely used in a paprika farm. Data for R1 is shown in Figures 4 and 5 for R2. The samples were taken to analyze the relationship in paprika ability after collecting the growth of leaves. The leaf is the independent variable and the dependent variable is the leaf's width, CO_2_, wind speed, dew point, humidity, and outside/inside temperature. This study has greenhouse climate variables that dataset correlated with warm summers and moderately cold winters. We calibrated paprika plant growth quality readings with a correlation between leaf growth, wind speed, dew point, input and output temperature, and CO_2_ [26]. This paprika growth data gets a more efficient leaf growth level in the autumn and winter season because of the temperature.

### 2.1. Data Preprocessing

The first step is to exclude all 0 entries from the paprika leaf growth and environmental variable tables. After this stage, the total number of entries was reduced to 48102. The next step is to exclude error data from the area of leaf count and environmental variables. The R1 and R2 plots of leaf and environmental variables are shown in Figures 4 and 5. The statistics show that both areas have many greenhouses, with a maximum of 3852 in the paprika leaf and a maximum of 48102 in the environmental variables. Getting rid of those outlier increases prediction accuracy. In all paprika leaf growth and energy variables data that is more than three standard deviations from the mean value is omitted.

### 2.2. Linear Classification

The simplest statistical classification approach for defining the linear relation between the independent and dependent variables is linear classification (LC) [27]. Fitting a linear equation line to the measured data is how it is done. It is critical to verify if there is a relationship between the variables or features of concern when fitting the model, which is done using the numerical variable, the correlation coefficient [28, 29]. The equation defines an LC line: *Y* = *a* + *b X*, the independent variable is *X*, while the dependent variable is *Y*. The “*b*” is the slope of the line and the “*a*” is the intercept (the value of *y* when *x* = 0). Its least square errors are widely used to determine the closest suited line, which is achieved by deducing the addition of squares of each point's vertical deviation from the line or the addition of squares of the residuals [30].

### 2.3. Random Forest

The random forest that can be used is caret R package both in the classification and regression model. The classification model refers to the factor/categorical dependent variables, and the regression model refers to the numeric or continuous dependent variable [31]. In random forest, we can include more data. It can perform well on a large database. The random forest gives a highly accurate output from the collection of decision trees [26]. Each decision tree draws the sample random data, and it predicts the accurate result at the end. It maintains efficient use of all predictive features.

### 2.4. Support Vector Machine

Based on statistical learning theory, Vapnik introduced SVM in the late 1960s [32]. SVM has achieved many state-of-the-art classifications. Accuracy outcomes for enterprise credit risk assessment. SVM is a form of supervised learning and is often used in classification and regression for data agglomeration and anomalousness detection. The SVM algorithm develops a model that increases the separation between data points in each collection with a tuning hyperplane. The SVM function in R package e1071 can be built as a model structure given in the testing and training dataset to predict the classification of supplemental data points. SVM is useful because it is quick and there is no danger of over-add-on the data. It provides accuracy even if the data is missing [26, 33].

### 2.5. Gradient Boosting Machine

In command to study a gradient boosting machine model in R studio, you will first have to install the gradient boosting machine library. The gradient boosting machine function requires you to specify certain statements, it will begin by qualifying the formula. This will include your response and forecaster variables. Next, will qualify the system of your response variable [26]. We specify if nothing then the gradient boosting machine will try to guess. Some commonly used distributions include “Bernoulli” logistic regression, “Gaussian” squared errors, “twist” t-distribution loss, and “poison” count outcomes. At last, we will specify the data and the ntree's statement [26]. By default, the gradient boosting machine model will assume 500 trees, which can provide a good estimate of our gradient boosting machine performance.

## 3. Results

Machine learning model SVM, RF, and GBM for the greenhouse paprika row planting (R1 and R2) focus on paprika growth production. We are analyzing the best-predicted R1 and R2 growth.

### 3.1. Significance Linear Classification Model

We conducted an origination analysis to find out which input and output parametric quantity have the highest applied confusion matrix correlation importance on the forecast of leaf growth during the training period from 2019 to 2020. In this study, the correlation, linear classification, and machine learning model SVM, RF, and GBM algorithms were used. The input parameters included leaf width and leaf growth, humidity, wind speed, dew point, CO_2_, and inside and outside temperature. The second association between energy requests and crop growth forms below. The greenhouse environment created the highest paprika correlation coefficients (*R*) and the lowest values of significance coefficients (Sig) and *P* values (*R* = 0.49 and Sig = 2.29 for R1 row planting and *R* = 0.62 and Sig = 3.27 for R2 row planting. Figures 6 and 7 show the pairs plot and display the correlation values of outdoor and indoor temperature, wind speed, dew point, CO_2_, and humidity. The dependent variable time interval has the lowest correlation value with the independent variables R1 and R2 row planting, with a maximum *R*-value of 0.99, as seen in the map. It used the linear classification procedure as an effective method to measure the result of all forecasters on greenhouse paprika. Internal temperatures and Carbon dioxide CO_2_ are the most important factor in the released greenhouse paprika according to scientific reasoning. The accuracy and kappa values were acquired by seeing all forecaster inputs values (R1 accuracy = 0.77 and kappa = 0.62 and R2 accuracy = 0.78 and kappa = 0.64 for passed off R1 and R2 row planting from energy, respectively). The results from the two characteristics R1 and R2 LC method, i.e., from this study, the paprika growth uptake was calculable to the best growth R2 more than R1.

The results from the linear classification model exposed almost related findings that the internal and the outside temperatures were the most important items on R1 and R2 row planting individually, except for the CO_2_ which was found to be valuable on the R1 and R2 row planting, a fact that was also according in other research papers in the literary study. In a visual perception of these collections, all input factors i.e., internal and outside temperatures, Carbon dioxide, humidity, dew point, and wind speed were chosen for the linear classification prognostic logical thinking of paprika growth.

### 3.2. Machine Learning Model

This study shows the statistical relationship metrics derived from the three ML models for the energy prediction time frame [34]. The findings reveal that RF outperforms all other ML models in terms of prediction times accuracy = 0.88. RF models can store information through their internal state records, which serve as long- and short-term databases, as shown by their narrow orbit of variability. When we impoverish to forecast new data sets on previous data sets, this capacity to store factual evidence is extremely useful. Equivalent to the technique results obtained by the LC model with this paper's location and data collection periods, the GBM model could have improved results with an accuracy of 0.85. The collection of SVM models affected well in the training phase but did not perform as well in the prediction phase accuracy = 0.84 and kappa = 0.66, respectively, and this is because of their low effectivity of the basic cognitive process in data series forecast tasks.

Analyzing models requires statistical validation, which is a crucial step. Following training, stratified 10-fold cross-validation was used to assess how well the three models performed. A statistical method that is frequently employed for assessing classification models is cross-validation. The dataset is divided into *k* folds, of which the *k* − 1 fold serves as the test data. The remaining folds are then sent to the models to serve as training data. The output average of each performance is then obtained after this procedure is repeated until all folds have been utilized as a training set. When working with fewer data, cross-validation is a wonderful technique to get more accurate findings [35].

### 3.3. Significance of Random Forest

In this article, the random forest CARET package in R studio is used to construct the paprika leaf and energy variables model based on the RF algorithm. Two tuning parameters, ntree 1700 to 1900 and mtry 1 : 15, must be set when creating this prediction model. The number of trees is represented by ntree. The smaller the fitting effect, the greater the ntree weight, and the value of ntree is often set to 1700, and the correlation between out-of-bag error and ntree size can be calculated [36, 37], as seen in Figures 8 and 9. If mtry denotes the set of feature attributes to be chosen, its value is usually the confusion matrix of all characteristic attributes. Since this paper has ten feature attributes, the accuracy bootstrap final values used for the model are R1 = 7 and R2 = 5.

Figures 8 and 9 show the results of the out-of-bag error and the validation error using the random forest model in R1 and R2. In the results, the green color reveals 0.046 class error, the black color has out of the bag 14.37% error, and the red color shows 0.28 class error when ntree is 500. When the out-of-bag error tends to be stable, its value is also low, then, the random forest model classification performance is higher. So, if we set the value of ntree to 1700 and the value of R1 mtry 15 and R2 mtry 15, we can train the original dataset of the first 3887 data and obtain the desired prediction model for the random forest congestion state. The remaining 122 sets of data were used as test data in the random forest model, and the R1 sets 7 and R2 sets 5 of data classification were used to arrive at the results depicted in Figures 10 and 11.

The accuracy rating shows that the classification of the right rate of reference is high, as seen in R2 in Figure 11. The random forest paprika leaf growth prediction model is accurate and can be used, as shown by the results in Tables 2 and 3. Furthermore, the random forest prediction model can compare R1 with R2 for the relative importance of energy causing congestion and determine the importance of environmental factors influencing the congested state. Figures 12 and 13 depict the findings. The energy efficiency of CO_2_ emissions was calculated as 91 percent. While this index is greater than 50 percent, we can find energy efficiency by using machine learning techniques to maximize stimulation.

### 3.4. Significance of Gradient Boosting Machines' Model

Machine learning models provide methods for calculating the aggregate influence of predictors on the model. The prediction accuracy on the out-of-bag portion of the data is recorded for each tree in boosted trees. Then, after permuting each predictor value, the process is repeated. The difference in accuracies is then averaged over all trees and normalized by the standard error. Grid search hyper-tuning parameter is used to select an approximately optimum configuration for each classifier. Based on an empirical study, the GBM model-specific tuning parameters resulted in the best accuracy models. The various grid searches were performed to identify the best tuning settings for each model. In certain cases, just one or two parameters, the CARET package in Figures 14 and 15, were tuned. Models with a large dimensional hyper-parameter search space, such as, on the other hand, result in GBM model configurations being trained, as illustrated in Figures 14 and 15.

In Figures 14 and 15, the output object is a collection that contains details about the model and performance. Routine indexing can access this knowledge. Here, the minimum CV accuracy of R1 is 0.84, but the plot also shows that the CV error is already declining at 1500 trees. Then, the minimum CV accuracy of R2 is 0.82, but the plot also shows that the CV error is already declining at 1500 trees [38, 39].

For each observation, the prediction results of Figures 16 and 17 reveal the predicted value R1 case 3, prediction value is 1.335 to case 8, prediction value is 1.038 and R2 case 6, prediction value is 1.13 to case 11, prediction value is 2.02 this classifier model fit and the most influential variables driving predicted value. In the end, the authors compare the model to make predictions based on the GBM lime model. Simply uses the prediction function, as in most models; however, supply the number of trees to use. The model makes predictions based on the regression method. GBM model lime best value is R1 1.03 [35]. The accuracy for our test range is like our best GBM model's R1 accuracy of 0.86 and R2 accuracy of 0.85.

## 4. Significance of Support Vector Machine

SVM Linear basis kernel requires two tuning parameters for the model: sigma and cost. The classification penalty is regulated by cost, and the radial basis kernel parameter is sigma. The sigma parameter is 1 : 9, and the cost is 3,6,9. The grid search shown in Figures 18 and 19 identifies the best SVM linear classification tuning parameters, sigma (1), and cost (9).

The SVM model was verified using 10-fold cross-validation after being evaluated with several hyper-tuning parameter combinations. The authors meticulously tweaked two hyper-tuning parameters of the SVM model until the optimum accuracy rate was attained. The first is the linear kernel function. The second factor is the cost value, which varies from 0.1 for the highest regularization to 10 for the weakest. Cost's range had been examined with each kernel function. Figures 18 and 19 demonstrate a substantial difference in the performance of the SVM model with an SVM linear kernel vs increasing cost values ranging from 0.1 to 9 [35].

## 5. Discussion

This paper addresses the role of temperature in the plant health condition particularly affecting paprika growth using environmental variables in energy. We analyzed ML approach that can help smart farms in improving their energy or environmental temperature control relating to agricultural energy. When the solar energy increased, the inside temperature and dew point of the greenhouse increased as well as the CO_2_ uptake concentration also increased. The relative humidity decreased. Changes in atmospheric temperature with increased temperature were attributed to the high solar energy rate in the paprika leaf and decreased dew point in the paprika leaf during daylight hours and the solar energy pattern of the smart greenhouse has a powerful time part. Solar energy is lower throughout the year except in summer. Smart farm solar energy consumption begins to rise in May and is supported high up to September end. In this section, the statistical relation metrics for estimating the daily relationship between the presented paprika leaf growth, environmental factor, and energy under various input combinations using the three ML models SVM, RF, and GBM are shown in Tables 2 and 3. The estimated accuracy values differed among various input combinations and ML model types. Tables 2 and 3 present comparative analytics results between training and testing data of R1 and R2, respectively, row planting in a train and test value. The comparative study of three different supervised machine learning models (SVM, RF, and GBM) is done to predict the best paprika crop growth in the smart farm that can help farmers to grow crops more efficiently. In completion, we concluded that the paprika growth prediction using the leaf as the constant variable, dataset showed the best accuracy with random forest classifier with 88.32%.

The most significant research uses information from smart farms. A recent paper uses a different model of training to present a distinctive addition to the subject of classifying paprika growth. The review section has offered a well-described process for how they can produce superior findings when writing their papers. The presented models, although having rather amazing performances, are nevertheless unable to outperform or even come close to matching the results of some of the most recent relevant research. The authors choose to explore other diverse ways to improve the performances of the suggested models to push the limits of machine learning application in crop growth categorization.

This study, through comparative analytics using machine learning models, shows that the performance was better than stand-alone algorithms. For training and testing data, RF, which is assembled by environmental and solar energy, performed better than other machine learning classifiers. RF had the highest accuracy of 0.88 and GBM and SVM had an accuracy of 0.86 and 0.84, respectively. In this test RF, which is one of the ntree-based ensemble machine learning models can be used as a strong method for paprika growth prediction. With all meteorological correlativity among different weather factors as like input temperature, output temperature, wind speed, dew point, CO_2_, and humidity variables, RF models exhibited the best estimation accuracy during training accuracy = 0.88, precision = 0.83, recall = 0.70, f1-score = 0.74, kappa = 0.75 and testing accuracy = 0.82, precision = 0.79, recall train = 0.69, f1-score = 0.71, and kappa = 0.72, as compared to models with the complete error values. As shown in Table 3, estimated daily paprika growth accuracy values also differed among SVM, GBM, and RF models. SVM models (accuracy = 0.84, precision = 0.81, recall train = 0.64, f1-score = 0.75, and kappa = 0.66 during training; accuracy = 0.81, precision = 0.79, recall = 0.63, f1-score = 0.69, and kappa = 0.61 during testing) slightly outperformed GBM models (accuracy = 0.85, precision = 0.81, recall = 0.67, f1-score = 0.75, and kappa = 0.69 during training and accuracy- = 0.75, precision -0.72, recall = 0.65, f-score = 0.73, and kappa- = 0.48 during testing) under various input combinations, followed by RF models (accuracy = 0.88, precision = 0.83, recall = 0.70, f1-score = 0.74, kappa = 0.75, and testing accuracy = 0.82, precision = 0.79, recall train = 0.69, f1-score = 0.71, and kappa = 0.72.) Compared to the SVM model, the estimation accuracy of GBM and RF models increased by 17.4–29.9 pct, 11.7–23.9 pct, and 3.5–13.3 pct in terms of accuracy under various input combinations during training, while the corresponding values were 17.6–28.6 pct, 8.8–23.2 pct, and 2.1–5.6 pct, respectively [1]. Because of its advantage in modeling dynamic non-linear interactions between paprika growth and its environmental variables, the RF model was more suited for regular paprika growth estimation. We discovered that as the number of input variables decreased, the increase in estimation accuracy of RF and decreased GBM models, indicating that the two models were more useful and has more complex relationships between multivariate inputs and outputs occurred. In the research point, Figures 11, 15, and 19 show plots of regular paprika growth values determined by RF, GBM, and SVM models against their respective calculated values under the three input combinations. Machine learning models with full input variables had aureate data point prediction models with Carbon dioxide, humidity, wind speed, indoor and outdoor temperature, and dew point, as seen in Tables 2 and 3. Furthermore, under all three input combinations, GBM and RF models provided fewer dispersed paprika growth estimates than SVM models. To further explore the difference in the distribution of observed and estimated accuracy values of measured and estimated daily paprika growth by SVM, GBM, and RF models under the three input combinations in the testing stage are presented. The recall obtained from the proposed maximum accuracy and specificity, but RF also achieves 0.70% recall comparable to the proposed LC model, is the key distinction between train-test split and 10-fold cross-validation approaches. The hyper parameterization performed in the ML model can be seen in Tables 2 and 3. This includes the number of tuning parameters set to RF 1700 to 1900, GBM 9, 12, 15, and SVM 3, 6, 9, set as the activation function of the model.

Tables 2 and 3 show the outcome of the research, the authors use another assessment measure or technique that considers the evaluation train and test data. This approach produced a significant outcome that outperformed the accuracy rating of all prior studies. The authors use the set of hyper-tuning parameters for each model that would be utilized to construct a suggested model using hyper-tuning parameterization. Tables 2 and 3 exhibit the accuracy, precision, recall, f1-score, kappa, and specificity of the proposed model for SVM, RF, and GBM using 10-fold cross-validation [35].

The current work got remarkable results in terms of numerous statistical methodologies, as shown in Table 3, using the suggested model given in this paper's methodology section. The authors determined that RF, as determined by many statistical validations such as confusion matrix, accuracy, kappa, and sensitivity, was the best model that produce the most superior results when compared to all previous research that used the same dataset. The current work achieves an accuracy rate of 0.88 percent, which is greater than all prior tests and research that used solar energy data [35].

## 6. Conclusions

This research aims to find out a hyper-tuning parameters prediction ML model for paprika growth control with solar energy usage and environmental factors in the Korean paprika region. The suggested model is based on a machine learning model for fixing and reducing the feature selection obstacles by applying the correlation between paprika leaf growth and environmental factors. The suggested model uses smart farm datasets for experiments and statistical analyses. RF, SVM, and GBM models were used to forecast paprika growth through analysis of the correlation between energy usage and environmental factors in the production of paprika. As the results of the comparative prediction test using the three models, the multi-level RF with a faster computation speed and a higher prediction efficiency was chosen as a superior model to GBM and SVM models. In the experiments with the suggested model, it revealed that most of the environmental factors consume energy through the process of paprika production, while CO_2_ takes first place. To maximize the efficiency of environmental energy usage for paprika cultivation, it shows that matching the indoor and outdoor temperature to 32 degrees Celsius is recommended. Therefore, the proposed model can support efficient smart service mechanisms of H/W and S/W for a smart farm than the other models by achieving the highest accuracy of 0.88 pct. Because of its high precision, the strengthened RF model can be used to make management decisions about paprika production and to develop an advanced forecasting service such as controlling the growth rate of crops and energy usage for crop cultivation.

### 6.1. Nomenclature

Table 4 shows the abbreviations used in this paper to propose a crop growth prediction model based on machine learning using environmental and energy data for the growth of paprika in a greenhouse.

## Figures and Tables

**Figure 1:** A conceptual diagram of the relationship between components and energy in a smart farm.

**Figure 2:** IoT software modules for smart farm.

**Figure 3:** Smart farm solar energy data from 2019 to 2020.

**Figure 4:** Paprika growth consumption measurement variables that are correlated to R1 (a). Paprika growth consumption measurement variables that are correlated to R1 (b).

**Figure 5:** Paprika growth consumption measurement variables that are correlated to R2 (a). Paprika growth consumption measurement variables that are correlated to R2 (b).

**Figure 6:** Correlation of environmental variables R1.

**Figure 7:** Correlation of environmental variables R2.

**Figure 8:** R1 random forest out-of-bag error vs validation error.

**Figure 9:** R2 random forest out-of-bag error vs validation error.

**Figure 10:** R1 random forest classification accuracy cross-validation.

**Figure 11:** R2 random forest classification accuracy cross-validation.

**Figure 12:** R1 random forest variable importance.

**Figure 13:** R2 random forest variable importance.

**Figure 14:** R1 GBM classification accuracy cross validation.

**Figure 15:** R2 GBM classification accuracy cross validation.

**Figure 16:** R1 paprika growth for observations 8 (high paprika production observation) and 3 (low production observations) using lime.

**Figure 17:** R2 paprika growth for observations 11 (high paprika production observation) and 6 (low production observations) using lime.

**Figure 18:** R1 SVM classification accuracy cross-validation.

**Figure 19:** R2 SVM classification accuracy cross-validation.

**Table 1:** Smart farm data material and description.

Data variables	Measurement
Date	dd/mm/yyyy and time
Leaf	Number of pct
Leaf width	9.4 to 11.3 cm
CO_2_	Parts-per-million (ppm)
Internal temperature	18°C
Outside temperature	26°C
Dew point	Or (dew point temperature (°C))
Humidity	RHmean daily mean relative humidity [pct]
Wind speed	1.2 = 2.50 mph
Solar energy	kWh

**Table 2:** Crop growth and energy in the ML models performance prediction R1 result.

Models	Training data		Testing data	
	Accuracy	Kappa	Accuracy	Kappa
Random forest	0.85	0.65	0.83	0.63
Gradient boosting	0.86	0.70	0.82	0.63
Support vector machine	0.84	0.66	0.81	0.61

**Table 3:** Crop growth and energy in the ML models performance prediction R2 result.

Models	Training data		Testing data	
	Accuracy	Kappa	Accuracy	Kappa
Random forest	0.88	0.75	0.82	0.61
Gradient boosting	0.85	0.69	0.75	0.48
Support vector machine	0.84	0.66	0.72	0.40

**Table 4:** Abbreviations.

Abbreviation	Definition
LC	Linear classification
R1	Row planting R1
R2	Row planting R2
AI	Artificial intelligence
ML	Machine learning
GBM	Gradient boosting machine
SVM	Support vector machine
RF	Random forest
IoT	Internet of tanking
TS	Training selection
Sig	Significant coefficients
CO_2_	Carbon dioxide
ntree	Number of trees
mtry	Number of randomly sampled variables
OOB	Out of bag
CV	Cross validation
CARET	Classification and regression training
MICAZ	Microcontroller and transceiver
nesC	National electrical safety cord
TinyOS	Open-source, BSD- based operating system
MIB 250	cMebibyte (measurement used in computer data storage)
ADO NET	ActiveX data object
Pct	Percentage (%)
Mph	Miles per hour
H/W and S/W	Hardware/Software.

## Data Availability

The dataset used to support the findings of the study can be obtained from the first author or corresponding author upon request.
